This article has been retracted.

# Effects and Safety of Sacubitril/Valsartan for Patients with Myocardial Infarction: A Systematic Review and Meta-Analysis

**DOI:** 10.1155/2022/7840852

**Published:** 2022-01-05

**Authors:** Lang Liu, Xiaofang Ding, Yaxiang Han, Jianfeng Lv

**Affiliations:** ^1^General Hospital of Ningxia Medical University, Yinchuan City 750000, China; ^2^Affiliated RenHe Hospital of China, Three Gorges University Second Clinical Medical College of China Three Gorges University, Yichang City 443000, China

## Abstract

Patients who develop heart failure (HF) after an acute myocardial infarction (AMI) are at higher risk of adverse fatal and nonfatal outcomes. Studies have shown sacubitril/valsartan can further reduce the risk of cardiovascular death or hospitalization for heart failure by 20% compared with enalapril. At the same time, its tolerance and safety are better. However, the current evidence regarding the efficacy of sacubitril/valsartan in patients with heart failure after acute myocardial infarction is controversial. To assess the effect of sacubitril/valsartan on heart failure after acute myocardial infarction, we conducted a systematic review of the literature and a meta-analysis of existing randomized clinical trials. Meta-analysis of randomized controlled trails is used where data are collected from PubMed, the Cochrane library, Embase, and Web of Science. Data about sacubitril/valsartan were available from 5 studies. Forest plots showed that the sacubitril/valsartan group had a 299% higher value of sacubitril/valsartan to the control group (MD = 2.99%, 95% CI: 2.01, 3.96, *I*^2^ = 78%, *P* < 0.00001, Figure 2), and the difference was statistically significant. Forest plots showed that the sacubitril/valsartan group had a 531% lower value of LVEF to the control group (MD = −5.31%, 95% CI: −7.36, −3.26, *I*^2^ = 91%, *P* < 0.00001, Figure 2), and the difference was statistically significant. Forest plots showed that the sacubitril/valsartan group had a 133% lower value of NT-proBNP to the control group (MD = −1.33%, 95% CI: −1.54, −1.12, *I*^2^ = 96%, *P* < 0.00001, Figure 3). Forest plots showed that the sacubitril/valsartan group had a 49% lower risk of heart failure to the control group (MD = 0.49, 95% CI: 0.27, 0.89, *I*^2^ = 0%, *P*=0.02, Figure 3). The patients in experimental showed an obviously lower OR of MACE (OR = 0.47, 95% CI: 0.27, 0.82, *P*=0.007, Figure 3). The data were statistically significant. We have observed that for patients with heart failure after acute myocardial infarction, early administration of sacubitril/valsartan can significantly reduce the incidence of heart rate, left ventricular ejection fraction, NT-proBNP, and MACE. Our meta-analysis suggests that taking sacubitril/valsartan is relatively safe and effective, especially if started early after acute myocardial infarction.

## 1. Introduction

Acute myocardial infarction (AMI) refers to the rapid reduction or interruption of coronary blood supply caused by plaque rupture, thrombosis, or coronary artery spasm on the basis of atherosclerosis, resulting in sustained and severe acute ischemia of the corresponding myocardial tissue and eventually lead to heart muscle cell death disease [1]. In the absence of timely and effective vascular opening, patients die within a short period of time from malignant arrhythmias, acute heart failure, cardiac rupture, and cardiogenic shock. In recent years, due to the continuous expansion of chest pain centers in China, the mortality rate of AMI patients is significantly lower than before [2]. Although emergency PCI can revascularize and save part of dying and damaged myocardium, some patients could still experience left ventricular remodeling postmyocardial infarction [3,4]. Ventricular remodeling includes myocardial hypertrophy, interstitial fibrosis, increased cardiac volume, and reduced diastolic function. LV systolic dysfunction caused by postacute myocardial infarction caused the sympathetic nervous system (SNS) increased excitability, and overactivation of the rennin-angiotensin-aldosterone system (RAAS) promotes the release of norepinephrine (NE), angiotensin II (II), aldosterone, endothelin, and other vasoconstrictor substances in the circulatory system. At the same time, the secretion of the natriuretic peptide system (NPS) synthesized by cardiomyocytes themselves to counter the action of the above active substances is absolutely insufficient or relatively insufficient, resulting in neurohumoral regulation disorder imbalance, acute hemodynamic disorders, and ultimately heart failure [5]. Therefore, early postoperative application of angiotensin-converting enzyme (ACEI) inhibitors or angiotensin receptor blockers, *β*-blockers, and mineralocorticoid antagonist has shown to reduce the risk of developing HF and death in patients at high risk of developing HF after MI is important [6–12].

Sacubitril/valsartan is an inhibitor of angiotensin II receptor enkephalinase (ARNI). It is composed of angiotensin II receptor blocker (ARB) valsartan and enkephalin inhibitor (NEPI) precursor AHU377 in a 1 : 1 ratio [13]. On the one hand, valsartan can block angiotensin type 1 receptor (AT1), inhibit the release of Ang II dependent aldosterone, and antagonize RAAS. It is beneficial to slow down the development of heart failure by reducing sympathetic nerve excitability and myocardial oxygen consumption, improving hemodynamics, and inhibiting myocardial fibrosis [14]. On the other hand, the degradation of natriuretic peptide system by enkephalinase (NEP) was inhibited by sacubitril, thus enhancing the natriuretic peptide system. For the atrial natriuretic peptide (ANP), brain natriuretic peptide (BNP), and C-type natriuretic peptide (CNP) system, NPS mainly mediates sodium excretion, diuresis, vasodilation, antagonism against RAAS, and inhibition of aldosterone secretion by activating membrane-bound NPS receptor and its second messenger loop guanosine monophosphate (cGMP) [15]. Animal experiments have shown that [16] ANP inhibits aldosterone-mediated myocardial fibrosis and has the effects of sodium excretion, diuresis, vasodilation, and heart protection. According to the guidelines for the diagnosis and treatment of acute and chronic heart failure published in ESC in 2016 [17], ARNI was recommended to replace ACEI/ARB in the treatment of heart failure patients.

After the publication of the primary results of PARADIGM-HF (prospective comparison of angiotensin receptor-neprilysin inhibitor with ACE inhibitor to determine impact on global mortality and morbidity in heart failure), a series of subsequent prespecified and post hoc analyses have provided detailed insight into the clinical and quality of life benefits of sacubitril/valsartan compared to enalapril [11,18]. However, in the latest results of the PARADISE-MI trial (prospective angiotensin receptor-neprilysin inhibitor versus ACE inhibitor trial to determine superiority in reducing heart failure events after MI), sacubitril/valsartan has aroused wide academic discussion. The efficacy of sacubitril/valsartan in acute myocardial infarction has not been clearly defined, so a large number of clinical trials have been carried out and achieved certain results.

In this study, we comprehensively searched and systematically evaluated the randomized controlled trials of sacubitril/valsartan in acute myocardial infarction, providing further evidence-based medical evidence for the clinical application of sacubitril and valsartan in acute myocardial infarction. We have observed that for patients with heart failure after acute myocardial infarction, early administration of sacubitril/valsartan can significantly reduce the incidence of heart rate, left ventricular ejection fraction, NT-proBNP, and MACE. Our meta-analysis suggests that taking sacubitril/valsartan is relatively safe and effective, especially if started early after acute myocardial infarction.

The remaining sections and contents are organized as follows. In subsequent section, proposed methods along with an efficient search method, which is utilized during the proposed study, is described in detail. In Section 3, experimental results and observations were discussed along with various issues with the existing state of the art approaches. Finally, concluding remarks along with sufficient future directions are provided.

## 2. Proposed Methods

### 2.1. Search Strategy

This meta-analysis was performed according to the Preferred Reporting Items for Systematic Reviews and Meta-Analyses (PRISMA) guidelines. PubMed, Cochrane library, Embase, and Web of Science were used to retrieve all relevant articles with the search terms LCZ696, sacubitril/valsartan, entresto, neprilysin inhibitor, and myocardial infarction. The references of the initial identified literatures were also screen to identify other relevant articles. The literature search was restricted to English language. Patients or the public were not involved in our research.

### 2.2. Study Selection and Data Extraction

Selection criteria of various studies are as follows: studies including patients with myocardial infarction, studies in the experimental group including patients administered sacubitril/valsartan, randomized clinical trials are included, and studies with eligible outcomes.

Exclusion criteria are as follows: we excluded those studied where randomized control trials are not available and absence of efficacy data and increase in heterogeneity was questionable. For multiple publications that were identified reporting on the same clinical study, the one with the most complete publication data was eligible. Any discrepancies were resolved by discussion. Detailed reviews of full-text articles on research design, baseline characteristics, outcomes, and toxicity were completed by Lang Liu and Peng Bao independently. The publication year, author's name, study design, number of patients, median age, abruption, antepartum hemorrhage, perinatal death, and preterm preeclampsia were reported in the articles, and Supplementary Materials were obtained from each included study (Table 1).

### 2.3. Quality Assessment

We assessed the quality of the included literature using the risk of bias in the Cochrane Collaboration. These areas include sequence generation, allocation hiding, blinding, incomplete result data, selective result reporting, and other sources of bias. The risk of bias in each study was classified as high, low, or unclear. We resolve any differences by consensus.

### 2.4. Statistical Analyses

For the statistical analysis, we have used the Review Manager 5.3 software (The Cochrane Collaboration; Copenhagen, Denmark). Continuous outcomes were expressed as standard mean differences (SMDs) or mean differences (MDs) with 95% confidence intervals (95% CIs). Dichotomous outcomes were expressed as risk ratio (OR) with 95% confidence intervals (95% CIs). Chi-square-based Q-tests and *I*^2^ statistic were assessed to the heterogeneity among studies. If *P* values <0.10 or *I*^2^ >50%, the random effects model was adopted to meta-analysis. Otherwise, the fixed effect model would be used. Sensitivity analysis was performed by omitting of any one study from the meta-analysis. Subgroup analysis for outcomes was also performed to explore the influencing factors.

## 3. Results

The baseline characteristics of the 5 eligible studies are given in Table 1. 1012 relevant articles were identified by eligible studies, characteristics literature search, and review of reference lists. After screening and eligibility assessment, we included in the systematic review and meta-analysis a total of 5 clinical trials involving the group of patients treated with sacubitril/valsartan and the control treatment (Figure 1).

### 3.1. LVEF and Heart Rate

Data about sacubitril/valsartan were available from 5 studies. Forest plots showed that the sacubitril/valsartan group had a 299% higher value of sacubitril/valsartan to the control group (MD = 2.99%, 95% CI: 2.01, 3.96, *I*^2^ = 78%, *P* < 0.00001, Figure 2), and the difference was statistically significant.

Data about sacubitril/valsartan were available from 2 studies. Forest plots showed that the sacubitril/valsartan group had a 531% lower value of sacubitril/valsartan to the control group (MD = −5.31%, 95% CI: −7.36, −3.26, *I*^2^ = 91%, *P* < 0.00001, Figure 2), and the difference was statistically significant.

### 3.2. NT-proBNP, HF, and MACE

Data containing the value of NT-proBNP were available from 4 studies. According to our results, forest plots showed that the sacubitril/valsartan group had a 133% lower value of NT-proBNP to the control group (MD = −1.33%, 95% CI: −1.54, −1.12, *I*^2^ = 96%, *P* < 0.00001, Figure 3), and the difference was statistically significant.

Data containing heart failure data were available from 3 studies. According to our results, forest plots showed that the sacubitril/valsartan group had a 49% lower risk of heart failure to the control group (MD = 0.49, 95% CI: 0.27, 0.89, *I*^2^ = 0%, *P*=0.02, Figure 3), and the difference was statistically significant.

Data were available from 3 studies. The patients in experimental showed an obviously lower OR of MACE (OR = 0.47, 95% CI: 0.27, 0.82, *P*=0.007, Figure 3). The data were statistically significant.

### 3.3. Publication Bias

We have conducted a publication bias test on 5 articles, and the test results prove that there is a certain publication bias. For patients with heart failure after acute myocardial infarction, early administration of sacubitril/valsartan can significantly reduce the incidence of heart rate, left ventricular ejection fraction, NT-proBNP, and MACE. Our meta-analysis suggests that taking sacubitril/valsartan is relatively safe and effective, especially if started early after acute myocardial infarction.

## 4. Discussion

With the understanding of the concept of early myocardial reperfusion and the maturity of interventional techniques, the nosocomial mortality of AMI is significantly reduced, but ARIC studies show that the incidence and mortality of HF after myocardial infarction are still very high [19]. Even after successful PCI, 30% of patients still experienced ventricular remodeling 6 months after surgery, increasing the risk of HF and death after myocardial infarction. Therefore, prevention and reversal of ventricular remodeling to reduce the risk of death or rehospitalization in patients with heart failure after MI is the main therapeutic goal. The results of this retrospective analysis indicated that the effects of sacubitril/valsartan and enalapril were similar, and the LVEF of the experimental group was significantly higher than that of the control group after treatment, indicating that sacubitril/valsartan effectively improved left ventricular function, which was consistent with the results of the PARADIGM-HF trial [20]. Previous EVALUATE-HF study showed that [21] oral administration of sacubitril/valsartan significantly improved ventricular remodeling compared with oral administration and enalapril. Ventricular remodeling is an important pathophysiological basis of heart failure after myocardial infarction. After the occurrence of acute myocardial infarction, the human body automatically activates the sympathetic nervous system and the RAAS system to increase blood volume, improve myocardial contractility, and enhance the pumping function of the heart, so as to achieve normal blood supply to the heart [22]. RAAS can be divided into the cyclic RAAS pathway and organization RAAS pathway [23]. The former affects the sodium metabolism and arterial compliance to regulate arterial pressure and has short-term effects on pathophysiology [24]. The latter has long-term effects [25], converting angiotensin I to angiotensin II. Angiotensin II secretion promotes the growth of cardiomyocytes and blood vessels [26], increasing the amount of blood returning to the heart. However, after long-term secretion, the sympathetic nervous system will continue to be activated, and aldosterone is secreted in large quantities, accelerating the process of ventricular remodeling, increasing myocardial contractility, accelerating heart rate, water and sodium retention, and other changes. Increased heart rate may also worsen heart failure and is emerging as a new therapeutic target [27]. Patients with acute heart failure often have a higher basal heart rate than patients with chronic heart failure [28]. Previous studies have shown that the incidence of all-cause death and readmission is significantly reduced in patients with acute heart failure if their heart rate decreases by more than HR 27 during hospitalization. At the same time, it is suggested that clinical stability and discharge are the key stages of heart rate control, and heart rate should be closely monitored and controlled [29]. Although heart rate control in patients with acute heart failure can be beneficial, rate control in clinical practice centers is unsatisfactory. A European study showed that although >80% patients were treated with beta-blockers, only <25% of patients reached the target dose, and <50% patients with acute heart failure reached the target heart rate (<70 beats/min) before discharge [30], limits the benefit patients can get from controlling their heart rate. The results of this analysis showed that the heart rate of the experimental group was significantly lower than that of the control group. Therefore, sacubitril/valsartan can safely and effectively reduce the heart rate of patients with acute decompensated heart failure.

Second, the results of this retrospective analysis showed that the NT-proBNP decreased significantly after the treatment of sacubitril/valsartan, and the experimental group was superior to the control group, suggesting that sacubitril/valsartan were safe and effective in the treatment of AMI with cardiac insufficiency. Coincidentally, it is consistent with the results of PIONEER-HF experimental study [31,32]. BNP and NT-proBNP are neuroendocrine hormones secreted by the heart, which have been proved to be important indicators for clinical diagnosis, treatment, and prognosis of patients with heart failure [33,34]. BNP was first isolated from pigs and subsequently found to be mainly synthesized in ventricles. Its concentration can change with ventricular wall tension and has a negative feedback regulating effect on ventricular filling pressure, so it has become an important biomarker. ProBNP is a precursor of BNP, an amino acid polypeptide, found in heart muscle cells. The gene transcription of BNP is induced by stretching the myocardial wall, such as ventricular remodeling, resulting in the lysis of proBNP into two fragments, namely, NT-proBNP and active BNP fragments. Active BNP can cause a series of responses to ventricular dilation, such as natriuretic, diuretic, vasodilator, inhibition of renin, and aldosterone secretion [35]. At the same time of the occurrence of AMI, the BNP synthesis gene of the living cells around the infarct area and the cells in the noninfarct area rapidly transcribed mRNA, and the increase of ventricular volume load further induced the overexpression of mRNA, and BNP was rapidly synthesized and released into blood. BNP has a half-life of about 20 minutes, while NT-proBNP has a half-life of about 60–120 minutes, which is more stable than BNP [36]. Therefore, NT-proBNP plays an important role in evaluating the size of myocardial infarction, the therapeutic effect of myocardial cell reperfusion, and the prediction of late myocardial remodeling [18]. Large-scale clinical studies [37–39] showed that in STEMI and NSTEMI patients, plasma levels of BNP and NT-proBNP at admission were positively correlated with the incidence of subsequent adverse events such as death from all causes, recurrent myocardial infarction, rehospitalization, and prolonged hospital stay. MACE in patients with acute myocardial infarction after PCI will seriously threaten their life, health, and quality of life, and accurate prediction of the risk of MACE after PCI is conducive to early adoption of corresponding prevention and control measures, so as to reduce the occurrence of MACE and ensure good outcomes of patients [40]. Our analysis showed that the incidence of MACE was lower in the observation group than in the control group after treatment with sacubitril/valsartan.

The limitations of this study are as follows: the overall quality of the literature is not high, and the sample size is small; due to the quality of the articles, some literatures did not specify specific random methods; some literatures did not specify the specific use of Western medicine for conventional treatment and only limited the drugs recommended by the guidelines; meanwhile, differences in subjects' age and concomitant diseases may increase the clinical heterogeneity between studies; and high clinical costs of sacubitril/valsartan.

Therefore, we demonstrated that sacubitril/valsartan sodium tablets can inhibit ventricular remodeling after acute myocardial infarction, improve cardiac function, reduce the incidence of adverse cardiovascular events, the rate of rehospitalization and mortality after myocardial infarction, and improve disease prognosis without significant adverse reactions. However, due to the limitations of the quality and quantity of the included literature and the risk of bias, its efficacy will be overevaluated, which needs to be further confirmed by big data and high-quality prospective randomized controlled studies to provide higher evidence-based medical evidence.

## 5. Conclusion and Future Directives

To assess the effect of sacubitril/valsartan on heart failure after acute myocardial infarction, we conducted a systematic review of the literature and a meta-analysis of existing randomized clinical trials. Meta-analysis of randomized controlled trails is used where data are collected from PubMed, the Cochrane library, Embase, and Web of Science. Data about sacubitril/valsartan were available from 5 studies. Forest plots showed that the sacubitril/valsartan group had a 299% higher value of sacubitril/valsartan to the control group (MD = 2.99%, 95% CI: 2.01, 3.96, *I*^2^ = 78%, *P* < 0.00001, Figure 2), and the difference was statistically significant. Forest plots showed that the sacubitril/valsartan group had a 531% lower value of LVEF to the control group (MD = −5.31%, 95% CI: −7.36, −3.26, *I*^2^ = 91%, *P* < 0.00001, Figure 2), and the difference was statistically significant. Forest plots showed that the sacubitril/valsartan group had a 133% lower value of NT-proBNP to the control group (MD = −1.33%, 95% CI: −1.54, −1.12, *I*^2^ = 96%, *P* < 0.00001, Figure 3). Forest plots showed that the sacubitril/valsartan group had a 49% lower risk of heart failure to the control group (MD = 0.49, 95% CI: 0.27, 0.89, *I*^2^ = 0%, *P*=0.02, Figure 3). The patients in experimental showed an obviously lower OR of MACE (OR = 0.47, 95% CI: 0.27, 0.82, *P*=0.007, Figure 3). The data were statistically significant. We have observed that for patients with heart failure after acute myocardial infarction, early administration of sacubitril/valsartan can significantly reduce the incidence of heart rate, left ventricular ejection fraction, NT-proBNP, and MACE. Our meta-analysis suggests that taking sacubitril/valsartan is relatively safe and effective, especially if started early after acute myocardial infarction.

## Figures and Tables

**Figure 1:** Forest plots of flow diagram.

**Figure 2:** Forest plots of LVEF and heart rate.

**Figure 3:** Forest plots of NT-proBNP, HF, and MACE.

**Table 1:** Baseline characteristics of included studies.

Author	Year	Disease	No. of exp.	No. of con.	Age of exp.	No. of con.	Sex of exp. (M/total)	Sex of con. (M/total)	Intervention (exp.)	Intervention (con.)
Chi Chen	2021	Acute myocardial infarction	42	39	51.28 ± 6.27	51.3 ± 6.21	27/42	24/39	Sacubitril/valsartan	Bisoprolol

Kieran F. Docherty	2021	Myocardial infarction	47	46	61.8 ± 10.6	59.7 ± 10.1	42/47	43/46	Sacubitril/valsartan	Valsartan

Ahmed Rwzq, MD. PHD.	2020	ST-segment elevation myocardial infarction	100	100	52 ± 9.2	57 ± 11.6	86/100	88/100	Sacubitril/valsartan	Ramipril

Haiyan Wang	2020	Acute anterior wall myocardial infarction	68	69	59.13 ± 7.15	60.56 ± 7.62	52/68	54/69	Sacubitril/valsartan	Enalapril

Yi Zhang	2020	ST-elevation myocardial infarction	79	77	60.3 ± 11.7	60 ± 10.9	59/79	55/77	Sacubitril/valsartan	ACEI

## Data Availability

The datasets used during the current study are available from the corresponding author upon request.

## References

[1] Arslan F., Bongartz L., Berg J. M. (2017). ESC guidelines for the management of acute myocardial infarction in patients presenting with ST-segment elevation:comments from the Dutch ACS working group. *Netherlands Heart Journal Monthly Journal of the Netherlands Society of Cardiology&the Nethe-rlands Heart Foundation*.

[2] Huo Y. (2014). Promoting chest pain center accreditation is an essential way to improve the management of acute myocardial infarction in China. *. Zhonghua xin xue guan bing za zhi*.

[3] Marek, Magdalena K.-W., Maciej W. (2018). Left ventricular reverse remodeling in patients with anterior wall ST-segment elevation acute myocardial infarction treated with primary percutaneous coronary intervention.. *Postepy w kardiologii interwencyjnej = Advances in interventional cardiology*.

[4] van der Bijl P., Abou R., Laurien G. (2020). Left ventricular remodelling after ST-segment elevation myocardial infarction: sex differences and prognosis. *. ESC heart failure*.

[5] Greco, Rosato S., D’Errigo P., Mureddu G. F, Lacorte E., Seccareccia F. (2015). Trends in mortality and heart failure after acute myocardial infarction in Italy from 2001 to 2011. *International Journal of Cardiology*.

[6] Pfeffer Marc A., Braunwald E., Moyé lemuel A. (1992). Effect of captopril on mortality and morbidity in patients with left ventricular dysfunction after myocardial infarction:results of the survival and ventricular enlargement trial. *New England Journal of Medicine*.

[7] Dargie H. J. (2001). Effect of carvedilol on outcome after myocardial infarction in patients with left-ventricular dysfunction: the CAPRICORN randomised trial. *The Lancet*.

[8] Zannad, Gheorghiade M., Henry K., Chu T.-C., Patni R., Pitt B. (2004). The effect of eplerenone on all-cause mortality and heart failure hospitalization in the eplerenone post-acute myocardial infarction heart failure efficacy and survival study (EPHESUS). *Journal of Cardiac Failure*.

[9] The Acute Infarction Ramipril Efficacy (AIRE) Study Investigators (1993). Effect of ramipril on mortality and morbidity of survivors of acute myocardial infarction with clinical evidence of heart failure. *Clinical Trail*.

[10] Køber L., Torp-Pedersen C., Carlsen J. E. (1995). A clinical trial of the angiotensin-converting-enzyme inhibitor trandolapril in patients with left ventricular dysfunction after myocardial infarction. Trandolapril Cardiac Evaluation (TRACE) study group. *The New England journal of medicine*.

[11] Robin A. P., Weir P. B. M., Petrie C. J. (2009). Left ventricular remodeling after acute myocardial infarction: does eplerenone have an effect?. *American Heart Journal*.

[12] Scott S., Karen P., Reed S. (2006). The effect of valsartan, captopril, or both on atherosclerotic events after acute myocardial infarction: an analysis of the Valsartan in Acute Myocardial Infarction Trial (VALIANT).. *Journal of the American College of Cardiology*.

[13] McMurray J. J. V., Packer M., Desai A. S. (2014). Angiotensin–neprilysin inhibition versus enalapril in heart failure. *New England Journal of Medicine*.

[14] Toru, Nakamura K., Miura D. (2019). Effect of LCZ696, a dual angiotensin receptor neprilysin inhibitor, on isoproterenol-induced cardiac hypertrophy, fibrosis, and hemodynamic change in rats. *. Cardiology journal*.

[15] Schoenfeld, West T., Verghese P. B. (2017). The effect of angiotensin receptor neprilysin inhibitor, sacubitril/valsartan, on central nervous system amyloid-*β* concentrations and clearance in the cynomolgus monkey. *Toxicology and Applied Pharmacology*.

[16] Nakagawa H., Heike O., Nikolaev Viacheslav O. (2014). Atrial natriuretic peptide locally counteracts the deleterious effects of cardiomyocyte mineralocorticoid receptor activation. *. Circulation. Heart failure*.

[17] Ponikowski, Voors A. A., Anker S. D. (2016). ESC guidelines for the diagnosis and treatment of acute and chronic heart failure. *Revista Española de Cardiología*.

[18] Docherty Kieran F., Muthiah V., Solomon Scott D. (2020). McMurray john J V. Sacubitril/valsartan: neprilysin inhibition 5 Years after PARADIGM-HF. *JACC. Heart failure*.

[19] Qureshi T., Zhang Z.-M., Chang P. P. (2018). Silent myocardial infarction and long-term risk of heart failure. *Journal of the American College of Cardiology*.

[20] McMurray John J. V., Milton P., Desai Akshay S. (2013). Dual angiotensin receptor and neprilysin inhibition as an alternative to angiotensin-converting enzyme inhibition in patients with chronic systolic heart failure: rationale for and design of the Prospective comparison of ARNI with ACEI to Determine Impact on Global Mortality and morbidity in Heart Failure trial (PARADIGM-HF). *. European journal of heart failure*.

[21] Desai S., Scott D., Solomon A. M. S. (2019). Effects of sacubitril-valsartan compared with enalapril on arterial hemodynamics, cardiac remodeling, and quality of life in patients with heart failure and reduced ejection fraction. *Journal of Cardiac Failure*.

[22] Schmidt M., Mansfield Kathryn E., Krishnan B. (2017). Adherence to guidelines for creatinine and potassium monitoring and discontinuation following renin-angiotensin system blockade: a UK general practice-based cohort study. *BMJ open*.

[23] Park K., Gaze David C., Collinson Paul O., Marber Michael S. (2017). Cardiac troponins: from myocardial infarction to chronic disease. *Cardiovascular research*.

[24] Liao, Chen K., Dong X. (2018). Berberine inhibits cardiac remodeling of heart failure after myocardialinfarction by reducing myocardial cell apoptosis in rats. *Experimental and Therapeutic Medicine*.

[25] (2018). ats. *Frontiers in Physiology*.

[26] Zullo R., Sadia S., Yoojin Lee M. S. (2017). Secondary prevention medication use after myocardial infarction in U.S. Nursing home residents. *Journal of the American Geriatrics Society*.

[27] Patrizio, Arnaud A., Julien M., Giovanni F., Piérard Luc A. (2015). Elevated heart rate at 24-36h after admission and in-hospital mortality in acute in non-arrhythmic heart failure. *International Journal of Cardiology*.

[28] Luigi, Michele S., Marco M. (2013). Multicenter prospective observational study on acute and chronic heart failure: one-year follow-up results of IN-HF (Italian network on heart failure) outcome registry. *Circulation. Heart Failure*.

[29] Takahama, Yokoyama H., Kada A. (2013). The extent of heart rate reduction during hospitalization using beta-blockers, not the achieved heart rate itself at discharge, predicts the clinical outcome in patients with acute heart failure syndromes. *Journal of Cardiology*.

[30] Farmakis, Parissis J., Karavidas A. (2015). In-hospital management of acute heart failure: practical recommendations and future perspectives. *International Journal of Cardiology*.

[31] Velazquez Eric J., Morrow David A., DeVore Adam D. (2019). Angiotensin-neprilysin inhibition in acute decompensated heart failure.. *New England Journal of Medicine*.

[32] Morrow A., Velazquez E. J., DeVore A. D. (2019). Clinical outcomes in patients with acute decompensated heart failure randomly assigned to sacubitril/valsartan or enalapril in the PIONEER-HF trial. *Circulation*.

[33] Chow S. L., Maisel A. S., Anand I. (2017). Role of biomarkers for the prevention, assessment, and management of heart failure: a scientific statement from the American heart association. *Circulation*.

[34] Troughton R., Michael Felker G., Januzzi J. L. (2014). Natriuretic peptide-guided heart failure management. *European Heart Journal*.

[35] Kim -Na, Januzzi J. L. (2011). Natriuretic peptide testing in heart failure. *Circulation*.

[36] Jin Joo P., Choi D.-J., Chang-Hwan Y. (2014). Prognostic value of C-reactive protein as an inflammatory and N-terminal probrain natriuretic peptide as a neurohumoral marker in acute heart failure (from the Korean heart failure registry). *The American Journal of Cardiology*.

[37] Morrow David A., de Lemos James A., Sabatine Marc S. (2003). Evaluation of B-type natriuretic peptide for risk assessment in unstable angina/non-ST-elevation myocardial infarction: B-type natriuretic peptide and prognosis in TACTICS-TIMI 18.. *Journal of the American College of Cardiology*.

[38] Manenti Euler R. E., Bodanese Luiz C., Camey Suzi A., Polanczyk Carisi A. (2006). Prognostic value of serum biomarkers in association with TIMI risk score for acute coronary syndromes.. *Clinical Cardiology*.

[39] James K., Lindahl B., Siegbahn A. (2003). N-terminal pro-brain natriuretic peptide and other risk markers for the separate prediction of mortality and subsequent myocardial infarction in patients with unstable coronary artery disease: a global utilization of strategies to open occluded arteries (GUSTO)-IV substudy circulation. *ACC Current Journal Review*.

[40] Yuli Setianto B., Budi Hartopo A., Sukmasari I., Puspitawati I. (2016). On-admission high endothelin-1 level independently predicts in-hospital adverse cardiac events following ST-elevation acute myocardial infarction. *International Journal of Cardiology*.

